# Metagenomic Human Repiratory Air in a Hospital Environment

This article has been retracted.

**DOI:** 10.1371/journal.pone.0139044

**Published:** 2015-10-02

**Authors:** Yi Yu Lai, Yanming Li, Jidong Lang, Xunliang Tong, Lina Zhang, Jianhuo Fang, Jingli Xing, Meng Cai, Hongtao Xu, Yan Deng, Fei Xiao, Geng Tian

**Affiliations:** 1 Genomics and Synthetic Biology Center, Tsinghua University, Beijing, China; 2 Department of Respiratory and Critical Care Medicine, Beijing Hospital, Beijing, China; 3 School of Medicine, Tsinghua University, Beijing, China; 4 Department of Hospital Infection Control, Beijing Hospital, Beijing, China; 5 Department of Medicine Laboratory, Beijing Hospital, Beijing, China; 6 State key laboratory of precision measurement technology and instruments, Tsinghua university, Beijing, China; 7 Beijing Hospital, Beijing Institute of Geriatrics, Key Laboratory of Geriatrics, Ministry of Health, Beijing, China; Peking University, CHINA

## Abstract

Hospital-acquired infection (HAI) or nosocomial infection is an issue that frequent hospital environment. We believe conventional regulated Petri dish method is insufficient to evaluate HAI. To address this problem, metagenomic sequencing was applied to screen airborne microbes in four rooms of Beijing Hospital. With air-in amount of sampler being setup to one person’s respiration quantity, metagenomic sequencing identified huge numbers of species in the rooms which had already qualified widely accepted petridish exposing standard, imposing urgency for new technology. Meanwhile,the comparative culture only got small portion of recovered species and remain blind for even cultivable pathogens reminded us the limitations of old technologies. To the best of our knowledge, the method demonstrated in this study could be broadly applied in hospital indoor environment for various monitoring activities as well as HAI study. It is also potential as a transmissible pathogen real-time modelling system worldwide.

## Introduction

Owing to the first coining of the term in 1998[1] and first conducting of high-throughput sequencing in 2006[2], metagenomic has gained tremendous progress over the past decade. This new technology is in a postion of recovering over 99% of microorganisms which are missing from conventional culture-based techniques[3] and bypassed the need for isolation & laboratory cultivation of individual strains[4]. Such advantages greatly widen its applications into various fields, such as medicine, engineering, agriculture, sustainable development and ecology[5]. The randomness of shotgun sequencing ensures that many species of microorganisms that would be otherwise unnoticed by traditional methods will be represented by at least some small sequence segments [6]. The procurement of largely unbiased gene samples from all members of detecting communities becomes technically feasible[7]. Particularly, with recent technical improvements, metagenomics can detect pathogens at very low abundance and even perform directly from clinical samples[8] or single cells[9].

This appealing technology has also been applied in medical fields, such as investigation of novel species and strains[10–12], outbreaks [13,14] and complex diseases[15,16]. However, there are very few reports about unbiased detection of hospital airborne microorganisms.

Hospital-acquired infection (HAI), also termed nosocomial infection in medical literatures [17], develops in a hospital environment, such as one acquired by a patient during a hospital visit or one developing among hospital staff. In the United States, there are roughly 1.7 million HAIs with about 99,000 deaths each year[18]. Such situation is attributed to two categories of airborne transmissible microorgnisms: maliganant infectious pathogens and environmental opportunistic infectious microbes. The latter category affects immune compromised patients and employees substantially, although it is not so virulent as the former. These two categories of epidemiology deserve much attention and routine monitoring, since both could develop into leathal problems if ignored. Airborne infection control is directly related with building ventilation community[19], cleaning regimes[20] and adverse events[21].

From **Table 1**along the main routes of HAI transmission: contact and droplet transmission were only in a short distance and could be prevented by administration and hygienic system. Vehicle and vector transmission although in a long distance, could be shut out by a similar precaution. Only airborne transmission could stay in the air for a long period of time and travel in long distance, not easy to be stopped by administration and hygienic regimes. Proper way of detection airborne transmission thus becomes a critical point after other administration and hygienic regimes have been followed.

**Table 1:** Main routes of transmission for nosocomial infection.

Router	Description
Contact transmission	The most important and frequent mode of transmission is by direct contact.
Droplet transmission	Transmission occurs when droplets containing microbes from the infected person are propelled a short distance through the air and deposited on the host's body; droplets are generated mainly by coughing, sneezing, and talking, and during the performance of certain procedures, such as bronchoscopy.
Airborne transmission	Dissemination can be either airborne droplet nuclei (5 μm or smaller in size) of evaporated droplets in the air for long periods of time or dust particles containing the infectious agent. Microorganisms carried in this manner can be dispersed widely by air currents and may become inhaled by a susceptible host within the same room or over a longer distance from the source patient, depending on environmental factors; therefore, special air-handling and ventilation are required to prevent airborne transmission.
Common vehicle transmission	This applies to microorganisms transmitted to the host by contaminated items, such as food, water, medications, devices, and equipment.
Vector borne transmission	This occurs when vectors such as mosquitoes, flies, rats, and other vermin transmit microorganisms.

The widely-used regulatory airborne microorganism sampling method is comprised of sedimentation or settle plate’s method. It had long been written into industry and ISO standards. However, this passive non-volumetric method is imprecise by over-representing larger particles due to their rapid settling rate. It is inefficient for collection of small particles because air turbulence around a plate can affect the results and tiny particles may never settle down. Like some spores, the aerodynamics diameter is between 2–5 um. Especially for surface hydrophobin[22] and static electricity, settle-down takes years of time and cannot be captured by a relatively short period of exposure.

Beside above regulated petridish capture, there are various bioaerosol sampling methods as showed in **Table 2**[23]. Certain limitations exist for commonly used bioaerosol samplers, such as for most of the samplers, nonbiological environmental particles such as dust must be separated from bioaerosols prior to detection[24], the diluted nature of bioaerosol[25] etc. However, for hospital airborne microbe monitoring, fast pace and lower detection limit will be more urgent than those of sampling accuracy. Since malignant infectious pathogens could kill people in a very quick way. Other environmental pollutants, albeit very threatening to health, need quite long term to be effective and generally no immediate medical treatment available. This made bioaerosol method more fit for applying in hospital rather than those for environmental in-depth study. The limitation of bioaerosol sampling becomes not so critical if being setup into a widely distributed network.

**Table 2:** Major types of bioaerosol samplers[23].

Sampler	Example of device
Impactors and Sieve Samplers	Anderson impactor; SAS; Burkard sampler
Impingers	AGI–30; Shipe sampler; Midget, multi-stage and micro-impingers
Centrifugal Samplers	RCS; Aerojet cyclone
Filter Cassette	Glass fiber; Teflon filters; Polycarbonate

Considering future application convenience, we used an air sampler with 0.2*μ*m polytetrafluoroethene (PTFE) filter membrane to intercept all microorganisms in the airflow. It could be regarded as a simplified bioaerosol method. The advantage of this way to routine bioaerosol air sampling [26] or cyclone method [27] is that the filter paper is easy to handle and mail to far away metagenomic lab for sequencing. **Fig 1B** are two pieces of filter papers, one with 24 hour captured airborne particles and another is blank control. Just the naked eyes we could see some difference. If some of the spraying liquid which can display some malignant pathogen on the filter paper could be technically worked out, monitoring people could then quickly decide whether it is necessary to mail certain samples. Such advantages are quite important while establish a monitoring network. Since most of the sampling sites are actually not only lack metagenomic equipment, but also lack trained personals to handle complex monitoring devices or follow complicated protocols. Therefore, the robust and cost effective filter paper system become a feasible choice. And for a huge monitoring network, individual sampler accuracy is not so important as that of network distribution. Moreover, filter paper does not sacrifice the detection limits. There is a research report which made use of automobile AC filters[28] to sample for 16S rRNA sequence. This is another cost-effective way for establishing a monitoring network. Not quite fit for hospital indoor air due to variation of aircondition distribution in room, but proper for hospital automobile monitoring, one of the HAI transmission routes in **Table 1**.

**Fig 1:** Number of metagenomic recovered species for each group of microorganisms. a) sampling equipment, the soft tube connected to sampling head allows it to be easily fixed at any position, even could be put before the mouth. b) the sampling filter paper at Nov.6,2013. Left: blank; right: after work for 24 hours. c) Numbers of species and d) proportions of species number in each group of microbes in four rooms.

We set up 24-hour air-in quantity pass filters which mimic that of human daily respiration. Generally human normal respiratory minute volume at rest is 5–8 L/min. During light activities, it may be around 12 litres. For the hospital environment, possibly 8 L/min represents a typical respiratory minute volume. However, 8 L/min includes inhale and exhale at once. So we approximately use half amount for our continuous samplers. That is 4 L/min.

There are four types of rooms in the hospital we visited: Respiratory Intensive Care Unit (sym. as HX), Intensive Care Unit (sym. as ICU), Outpatient Hall (sym. as MZ), and Emergency (sym.as JZ). Except for Outpatient Hall, the other three rooms have routine quality control reports which qualify the conventional petridish exposure measurement standard. Regulations of this hospital require air-exposure of 9cm blood agar petridish for 5 min and then incubation of 24 hour for counting. The limitation is that the colony count after incubation will be ≤ 4 CFU/dish averaged from 3 repeats. If the sampling is within 2 hour after sanitation, the exposed time should be extended to 15 min. The Outpatient Hall lacks such reports but provides similar hygienic and sanitation procedures. The official reports from this hospital near our metagenomic sampling time points are shown in **S1 Table**. The reports indicate that this hospital is well qualified with such “regulated” standards like most hospitals in the world. However, under such “qualified” conditions, metagenomic technology still recover a huge number of microbial species, among which the list of pathogenic species is presented. Considering the high death rate of HAI[18] each year and that petridish exposure is a widely-accepted standard, we know that most HAI death cases occur in hospitals “qualified” with such regulated standards. The patients are living in the hospital rooms for a long time instead of exposed inside for a short time like we do with a petridish. Thus, we reasonably believe that the new sampling system is more close to a real condition than its conventional counterpart. And the feasible way to substantially reduce HAI death rate should possibly be widely application of metagenomic sequencing rather than conventional petridish exposuring method. This new system should be addressed with much attention and research work.

## Materials and Methods

### Ethics Statement

The experiments in this study were official approved by the Beijing Hospital.

### Air sampling

All samples were collected in Beijing Hospital (google LatLng Marker location: 39°54'3.5", 116°25'0.78"), details of the room conditions were listed in **Table 3**. We set up an air sampling pump (SKC,PA,US) and connected to a 47mm filter holder (PALL, NY,U.S.) by TYGON tube (Saint-Gobain Corporation,US), with a 47mm,0.2um PTFE Membrane filter (PALL, NY,U.S.) inside. **Fig 2A** shows the tube with the holder. All filters were sterilized by autoclaving following the user’s guide, then packaged in sterilized aluminum foil and stored in a sealed bag until loading into the filter holder. The holder and all the tools used for changing new filters were cleaned with 75% ethanol or autoclaved each time to avoid contamination. The air sampler was drawn at an average flow rate of 4 L/min for 24 h (4:00 PM to 4:00 PM the next day). The sampling day was December 20, a clear day without PM2.5 pollution outdoor. At that day PM2.5 = 30.3 PM10 = 42.5, lower than mean value of 2013 (PM2.5 = 89).

**Fig 2:** Rarefaction Curve for data effectiveness. Abscissa: number of reads, coordinate: number of species.

**Table 3:** Visiting hospital room condition and sampler position.

Sample	Room Area (m^2^)	Temperature(°C) and humidity	Visiting people	Sampler position
ICU	30	22°C, 30%	12 beds / room*	center, bed height
HX	20	22°C, 30%	6 beds / room*	center, bed height
MZ	200	22°C, 30%	5000 people/day	center, counter height
JZ	40	22°C, 30%	1300–1400 people/day	center, counter height

* At the time of sampling, all beds in ICU and HX were occupied by the patients.

### DNA Extraction and metagenomic amplification

Each membrane filter was carefully removed from the holder and cut into small pieces. The pieces were put into a 15 ml sterilized centrifuge tube, which was added with 1 ml of ddH_2_O. After vigorously vortexing for 1 hours, the ddH_2_O was transferred into a sterilized Eppendorf tube. Half go to Petri dish culture with blood agar and half go to metagenomic detection. (Blood agar generally fit for bacteria culture.) DNA was extracted according to the protocol of a MO-BIO PowerSoil DNA isolation mini-kit (Carlsbad, CA, U.S.). After elution into a 10 ul elution buffer, whole genome was amplified by a REPLI-g® Single Cell Kit (Qiagen, Hilden, Germany). Blank control samples were set by placing a sterilized filter inside the sampler without operation for 23 h, and treated similarly as above. The samples and blank control samples were sent into whole genome amplification on a realtime PCR machine StepOne (Life technologies, CA, U.S.). With the blank control as baseline, the sample is significantly amplified, and the efforts of blank control DNA library generation failed to generate useable sequencing libraries, indicating that there was no DNA or species contamination. All the extracted DNA samples were stored at −80°C until further use.

### Sequencing and Data Quality Control

All the DNA library was prepared following user’s manual of enzymatics (Enzymatics, MA, U.S.). Illumina HiSeq 2500 sequencing systems (Illumina, CA, U.S.) were used for sequencing. Sequencing library construction and template preparation were performed according to the enzymatics library preparation protocol. We constructed a paired-end library with insert size of ∼500 bp for each sample. An aliquot of 1 *μg* amplified DNA from each sample was used for library preparation, which ensured sample consistency. In order to minimize possible PCR-introduced bias, PCR amplification was performed in 12 cycles. Each sample was barcoded and equal quantities of barcoded libraries were used for sequencing. Data with adaptor contamination and low-quality reads were discarded from the raw data.

## Results and Discussion

Two parallel samples under same conditions for each site were separately sent to conventional petridish culture and metagenomic sequencing with Illumina Hiseq 1500. Due to the difficulty in culturing most Archaea and Viruses, and since Eukaryota include some non-fungi species undetectably by any pure culture technology, we only selected Bacteria as a recovering contrast of culture-based technology. With same blood agar plates for those of sanitation inspection in **S1 Table**. With efforts, the medical laboratory in the hospital cultured out some bacterial species from the air sample as listed in **Table 4**. The abundance data along with the petridish counting were determined from metagenomic measurement. The medical laboratory generally could identify species only to genus by 16s PCR and some experiences. Together with all the species relevant to those cultured genus in **Table 4**from our metagenomic list, totally there were 157 bacterial species in **S2 Table**. Even though, the number of cultured species was still a small portion of the total metagenomic bacterial species. Such great difference in recovering rate is due to methodology. It should be noted that some of these missing species were cultivable and did grow on blood agar. Cultivable species still fail to grow on blood agar. This means that the culture-based technology, although has been established and regulated quite long, was actually not sensitive enough for detection of unknown pathogen, even for cultivable and well known species. For the blank no DNA library could be constructed, which indicate no DNA or microorganism contamination on filter papers or inside our pump system.

**Table 4:** Results in bacteria comparative culture of parallel hospital samples (Filter paper elution half to metagenomic sequencing and half to conventional Peri dish culture).

date	room	species	Metagenomic Abundance	Counting (cfu/sample)
2013.12.24	ICU	Micrococcus luteus	17,653	6
	ICU	Bacillus	26,922	2
2013.12.24	JZ	Micrococcus luteus	485	18
	JZ	Staphylococcus	14,202	20
	JZ	Bacillus	3,554	13
	JZ	Corynebacterium	18,579	4
2013.12.25	HX	Bacillus	3,300	32
	HX	Staphylococcus sciuri	22	10
	HX	Acinetobacter baumannii	14,280	2

(For those not identified to species such as Bacillus, Genus abundance instead of species abundance was used).

With a pair-end sequencing strategy, we discarded the adaptor contamination and low-quality reads from the raw data and finally generated ~17, ~13, ~5, ~2 billion clean bases of sequence data from metagenomic DNAs derived from ICU, Respiratory, Outpatient and Emergency, respectively **Table 5**. For metagenomic analysis, all clean data were uploaded to MG-RAST (Metagenomic Analysis Server). Before analysis, the following sequences were removed: artificial replicate sequences produced by sequencing artifacts [29]; any host-specific species sequences (H.sapiens, NCBI v36) using DNA level matching with bowtie[30]; low quality sequences using a modified DynamicTrim[30], which specifies the lowest phred score (= 15) counted as a high-quality base and trims sequences to contain less than 5 bases.

**Table 5:** Processing of metagenomic sequencing data (clean data have been uploaded on Mg-rast).

Sample	Raw_reads	Raw_bases	Clean_reads	Clean_bases	Ratio
ICU	174,474,182	174474182101	173,728,752	17,546,603,952	99.57%
HX	128,418,162	12,970,234,362	128,133,412	12,941,474,612	99.78%
MZ	45,966,580	4,639,099,292	45,829,914	4,625,305,072	99.70%
JZ	21,335,980	2,153,106,418	21,229,302	2,142,349,120	99.50%

The sequencing data were analyzed by MG-RAST, a widely-used metagenomics data analysis pipeline. M5nr (M5 non-redundant protein database) was limited by a maximum e-value of 1e-5, a minimum identity of 60%, and a minimum alignment length of 15 measured in aa for protein and bp for RNA databases. **Fig 2**shows that the numbers of species in four rooms approximate to the plateau. The rarefaction curve (analyzed by MG-RAST 3.3) suggests that the sequencing depth of the HiSeq data is sufficient to capture most of the microorganisms.

The numbers of identified Archaea, Bacteria, Eukaryota and Virus species are 106 (3%), 2170 (52%), 1679 (40%) and 211 (5%), respectively, at ICU; 72 (2%), 1597 (46%), 1759 (50%) and 60 (2%), respectively, at Emergency; 98 (3%), 2261 (65%), 1025 (30%) and 81 (2%), respectively, at Outpatient; 74 (2%), 1826 (51%), 1580 (44%) and 117 (3%), respectively, at Respiratory ICU (**Fig 1B and 1C and Table 6**). **Fig 1A** shows the sampling equipment and **Fig 1B** shows the filter papers. For all four rooms, the proportion of Bacteria and Eukaryota species together exceeds 90%, while that of Archaea and Viruses species together is relatively small. The heatmap of Archaea, Viruses, top 100 Eukaryota species, and top 100 Bacteria species are shown in **Fig 3**. Relevant excel tables were loaded in **S1–S4 Excel Files**.

**Fig 3:** Heatmap of metagenomic recoverd species for each group of microorganisms in four rooms. For bacteria and eukaryote, top 100 abundant species for the heatmap.

**Table 6:** Numbers of metagenomic recovered species in four rooms.

	ICU	JZ	MZ	HX
Archaea	106	72	98	74
Bacteria	2,170	1,597	2,261	1,826
Eukaryota	1,679	1,759	1,025	1,580
Viruses	211	60	81	117

As showed in **Table 4**and **S2 Table**, the hospital laboratory only detected a part of pathogens, and the detected genera of *Staphylococcus*, *Bacillus and Corynebacterium* included some pathogen species. *Acinetobacter baumannii* is the only pathogen species directly detected by that laboratory. It becomes increasingly important as a source of nosocomial infection [31]. *A*.*baumannii* was identified by a European ICU as responsible for 19.1% of ventilator-associated pneumonia (VAP) cases [32].

However, even in the top 100 species of genomically abundant bacteria, some cultivable pathogens were still not detected although they had long been cultured by the medical laboratory. These pathogens and the diseases they induced are listed in **Table 7**, which indicates petridishes as an unstable tool for pathogen detection and also reflect the metagenomic robustness compared to the conventional counterpart. Those missing pathogens included published noncosomicol pathogen such as *Enterococcus faecalis*, *Klebsiella pneumonia*. They have higher infectious rates in hospital environment than in outdoor region. Also some severe pathogens such as *Neisseria* or *Salmonella* presented. *Propionibacterium acnes* is presented highest in all four rooms of the hospital, still failed to be screened by Petridish method. It is probably a hospital environment airborne indicative bacterial species.

**Table 7:** Reported pathogens among metagenomic recovered top 100 abundant bacteria species, missed by regulated culture-based technology from parallel control.

Species	Room and metagenomic abundance				Pathogen
	HX	ICU	JZ	MZ	
Bacteroides fragilis	4746	28371	3027	2149	opportunistic pathogens[33]
Enterococcus faecalis	2321	18330	778	6940	nosocomial pathogen[34]
Klebsiella pneumoniae	1517	7201	859	28847	nosocomial pathogen[35]
Moraxella catarrhalis	5077	12138	332	8075	human pathogen[36]
Neisseria gonorrhoeae	1636	4917	291	8304	pathogen of gonorrhea[37]
Neisseria meningitidis	4412	18817	942	32350	pathogen of meningitis[37]
Neisseria mucosa	2458	15238	189	15407	induce endocarditis[38]
Neisseria sicca	2371	23286	228	37762	opportunistic,pneumonia[39]
Propionibacterium acnes	84389	211447	40758	3920201	opportunistic pathogen[40]
Proteus penneri	1504	66	2	47	invasive pathogen,nosocomial[41]
Pseudomonas fluorescens	3841	5226	140	4011	opportunistic infection[42]
Salmonella enterica	3101	23220	762	66357	Salmonellosis[43]
Shigella sonnei	1301	22349	656	17619	pathogen of shigellosis[44]
Streptococcus sp.	3194	10863	956	664	pneumonia,many infections[45]

It is not surprised that some seawater species and Cyanobacteria are presented in the recovered list. However, what astounds us is that *Shewanella frigidimarina*, an Antarctic coldwater anaerobic species [46] is present in four rooms. Though we do not know how it traveled so far here, the powerful metagenomic sequencing with recovering capability shows its presence, not in one room but in all four rooms. If we were restricted to the petridish method, we cannot detect such trace species only from a piece of air filter membrane. This reminder the potential network monitor of this method due to the lower detection limit of which VS culture based technology and the easy handling of the system.

The Principal coordinates analysis (PCoA) (**Fig 4**) revealed the significant difference of the four rooms we sampled with the outdoor metagenomic sequencing results from other literature [47], indicating that the indoor airborne microorganism pattern is quite different with that of outdoor pattern. Only 36 species cross indoor air and outdoor air as in **S3 Table** [47] among thousands of species.

**Fig 4:** PCoA analysis for indoor and outdoor air. Data were normalized between 0 and 1 and compared with PM2.5 and PM10 data set[47]. (red: Indoor results; blue: outdoor results).

For the intersection of species in four rooms, we identified 39 Archaea, 1425 Bacteria, 412 Eukaryota and 12 Viruses. Various intersections are shown in **Fig 5**.

**Fig 5:** Species intersection of each group of microbes in four rooms.

Tree view reflects the genomic distance to some degree, although it is not the real evolution tree. We plotted the tree view for each group of microorganisms in four rooms as shown in **S1 Fig**. There might be some bases for further study the relationship of those species in hospital environment.

## Conclusions

This study demonstrates the impact of application of metagenomic technology in hospital indoor air for various monitoring as well as in-depth study. Metagenomic technology can easily screen out thousands of microorganisms or cells or genes in a few hours, which is far more rapid than the conventional culture-based method. The time efficiency, board spectrum and lower detection limit are advantages for metagenomic technology entering a regulatory auditing system. The sampling system in this study is composed of a head connected to a soft TYGON tube (**Fig 1A**). It can be very conveniently fixed into a specific position, such as a patient’s head on a bed, or even can be directly put before a patient’s mouth for study on aerosol-borne microganisms. This system can also detect uncultivable trace species, such as *Shewanella frigidimarina*. Therefore, monitoring a worldwide infectious disease will be feasible. Network arrangement of such easy operation and cost effective monitoring system is highly recommended and regulatory auditing standard is imperative for both application and research.

*Propionibacterium acnes* is presented highest in all four rooms of the hospital. It is probably a hospital environment airborne indicative bacterial species with high patient visiting rate. *Aspergillus fumigatus* is fungi speices presented highest in most rooms, as our other study demonstrated it was correlated with humidity, not visiting people.

## Supporting Information

S1 Fig Tree view of each group of microbes in four rooms. (DOC)

S1 Excel Files Excel file of metagenomic recovered species in HX room. (XLSX)

S2 Excel Files Excel file of metagenomic recovered species in ICU room. (XLS)

S3 Excel Files Excel file of metagenomic recovered species in JZ room. (XLSX)

S4 Excel Files Excel file of metagenomic recovered species in MZ room. (XLSX)

S1 Table Summary of hospital petridish exposing QA reports near the day with metagenomic sampling. (DOC)

S2 Table The bacteria species relevant with hospital cultured genera in parallel samples. (DOC)

S3 Table 36 species which intersected with the 48 species in PM 2.5 paper[46]. (DOC)
